#  Structural and functional comparison of fumarylacetoacetate domain containing protein 1 in human and mouse

**DOI:** 10.1042/BSR20194431

**Published:** 2020-03-04

**Authors:** Alexander K.H. Weiss, Andreas Naschberger, Elia Cappuccio, Christina Metzger, Lorenza Mottes, Max Holzknecht, Jill von Velsen, Matthew W. Bowler, Bernhard Rupp, Pidder Jansen-Dürr

**Affiliations:** 1 University of Innsbruck, Research Institute for Biomedical Aging Research, Rennweg 10, Innsbruck A-6020, Austria; 2 University of Innsbruck, Center for Molecular Biosciences Innsbruck (CMBI), Innrain 80-82, Innsbruck A-6020, Austria; 3 Medical University of Innsbruck, Division of Genetic Epidemiology, Schöpfstrasse 41, Innsbruck A-6020, Austria; 4 European Molecular Biology Laboratory, Grenoble Outstation, 71 Avenue des Martyrs, CS 90181, Grenoble 38042, France

**Keywords:** crystallography, FAHD1, SIRT3

## Abstract

FAH domain containing protein 1 (FAHD1) is a mammalian mitochondrial protein, displaying bifunctionality as acylpyruvate hydrolase (ApH) and oxaloacetate decarboxylase (ODx) activity. We report the crystal structure of mouse FAHD1 and structural mapping of the active site of mouse FAHD1. Despite high structural similarity with human FAHD1, a rabbit monoclonal antibody (RabMab) could be produced that is able to recognize mouse FAHD1, but not the human form, whereas a polyclonal antibody recognized both proteins. Epitope mapping in combination with our deposited crystal structures revealed that the epitope overlaps with a reported SIRT3 deacetylation site in mouse FAHD1.

## Introduction

The superfamily of fumarylacetoacetate hydrolase (FAH) proteins describes enzymes that share a conserved catalytic center, yet exhibit multifunctionality in prokaryotes and eukaryotes [1]. Whereas many distinct FAH superfamily members were described in prokaryotes [1], the only identified members in eukaryotes are FAH and FAH domain containing proteins 1 and 2 (FAHD1 and FAHD2) [1–3]. FAHD1 was identified as oxaloacetate decarboxylase (ODx), and as such acts as a regulatory enzyme in the TCA cycle; accordingly, as it was associated with the regulation of mitochondrial function [4,5].

This work describes the structure and kinetic profile of the mouse protein. The structural basis for the bifunctionally of the human protein, i.e., ODx and acylpyruvate hydrolase (ApH), was recently described [6]. In the current manuscript, structure and functionality of both mouse and human enzymes are compared. A rabbit monoclonal antibody (RabMab 27-1) could be produced that is able to recognize mouse FAHD1, but not the human form, whereas a polyclonal α-hFAHD1 (anti-human FAHD1) antibody recognized both proteins. Epitope mapping in combination with our deposited crystal structures revealed the epitope recognized by RabMab 27-1, which overlaps with a reported SIRT3 deacetylation site in FAHD1. Potential implications of these findings are discussed below.

## Materials and methods

### Cloning and protein expression

Cloning and expression followed a defined protocol [7]. Mouse FAHD1 cDNA (GenBank NP_075969) was inserted into the pET30a vector system (Merck, His6/S-double-tagged: MHHHHHHSSGLVPRGSGMKETAAAKFERQHMDSPDLGTM…) using restriction enzymes. The resulting expression vector was introduced into BL21(DE3) *Escherichia coli LysS* bacteria. Clones were obtained via streaking bacteria on LB agar plates using ampicillin/chloramphenicol selection. A single colony was picked, and an overnight culture was grown in 1000 ml NZCYM medium, containing the respective selective antibiotics. At 37°C the bacteria were amplified to an optical density of 0.4 at 600 nm. Protein expression was induced by the addition of 500 μM isopropyl-1-thio-β-d-galactopyranoside (IPTG) and incubation was continued for 4 h at 37°C. Bacteria were harvested via centrifugation and stored at −70°C.

### Enzyme purification

Enzyme purification of His6/S-double-tagged proteins followed a defined protocol [7]. Recombinant protein was extracted via a three-step purification strategy involving metal affinity chromatography (Ni-NTA), anion exchange chromatography, and gel filtration (SEC). Fractions containing FAHD1 were pooled, concentrated and stored at −70°C. Gel electrophoresis of two preparations followed by silver staining verified the protein’s homogeneity; contaminations were barely visible (<<100 ng/μl).

Recombinant mouse FAHD1 (mFAHD1) of concentration in between 1.5 and 2.0 mg/ml (Vivaspin 10 MWCO) was sent for high throughput screening at the HTX laboratory (EMBL, Grenoble). Native mFAHD1 and mFAHD1 supplemented with 1 mM oxalate were screened for crystallization, and hits were obtained in various conditions. A total of 68 crystals were harvested by laser photoablation, cryo-cooled using the CrystalDirect Robot [8,9], and screened for diffraction. Best diffracting crystals of mFAHD1 grew from 25% (w/v) PEG 3350, 0.2 M MgCl_2_ and 0.1 M Bis/Tris pH 5.5 and for the oxalate bound protein from 20% (w/v) PEG 4000, 0.05 M MgCl_2_ and 0.1 M MES pH 5.5. As the crystals were small needles with volumes between 10^−6^ and 10^−5^ mm^3^ a beam diameter of 15 μm was selected [10]. X-ray diffraction data were collected by the autonomous European Synchrotron Radiation Facility (ESRF) beamline MASSIF-1 [11–13] using automatic protocols for the location and optimal centring of crystals [14]. Strategy calculations accounted for flux and crystal volume in the parameter prediction for complete datasets. All data were processed using the automatic pipelines at the ESRF [15].

### Structure determination

After correcting for moderate diffraction anisotropy using *StarAniso* [16], the native and complexed structures were phased by molecular replacement using *Molrep* [17] with chain A of the hFAHD1 structure [6] (PDB: 6FOH) as search model. Native and complexed mFAHD1 crystallized in space group *P*2_1_ (No 4) with related cells containing four copies of mFAHD1 (two dimers) per asymmetric unit (ASU). Model building was carried out in *Coot* [18] followed by iterative cycles of real space and reciprocal space refinement in *Coot* [18] and *Refmac5* [19]. Local non-crystallographic (NCS) restraints were applied and each mFAHD1 molecule in the ASU was assigned a single TLS group. In late-stage model building, magnesium ions and oxalate ligands were placed into the difference electron density map and refined. A small twining fraction was observed for 6SBI, but no improvement of global statistics or map quality resulted from twin refinement. Despite substantial anisotropy and resulting low outer shell completeness, the models are of good quality with expected stereochemistry as validated during the PDB deposition [20]. Data collection and refinement statistics are summarized in Table 1. Structure figures were generated using *Pymol* [21] and *UCSF Chimera* [22].

**Table 1:** Crystallization, data collection, and refinement statistics summary for mFAHD1 crystals and structure models

**Crystallization and data collection**		
Protein	mFAHD1, native	mFAHD1–oxalate complex
Model (PDB identifiers)	Chains A, B, C, D in 6SBJ	Chain A, B, C, D in 6SBI
Protein stock solution	1.5–2.0 μg/μl, SEC quality	
Crystallization conditions	25% (w/v) PEG 3350, 0.2 M MgCl_2_ and 0.1 M Bis/Tris pH 5.5	20% (w/v) PEG 4000, 0.05 M MgCl_2_ and 0.1 M MES pH 5.5, 1mM Na-oxalate
Beam line, wavelength (Å)	ESRF MASSIF-1, 0.96598	
ESRF data identification link*	https://doi.esrf.fr/10.15151/ESRF-DC-186917546	https://doi.esrf.fr/10.15151/ESRF-DC-187128349
Crystal volume (mm^3^)	10^−6^ to 10^−5^	
Space group (number)	*P*2_1_ (4)	
Cell parameters (Å) Cell parameters (°)	52.40, 69.96, 107.56 90.0, 92.25, 90.0	52.60, 103.35, 86.60 90.0, 90.21, 90.0
Unit cell volume (Å^3^)	393781	470545
Solvent fraction, V_M_ (Å^3^/Da)	0.27, 1.68	0.39, 2.00
Wilson B-factor (Å^2^)	35.6	38
Resolution^1^ (Å) anisotropic (Å)	42.65-2.22 (2.47-2.22) 2.22, 2.37, 2.77	44.38-2.70 (2.97-2.70) 2.81, 3.93, 2.65
Completeness^1^, spherical elliptic (%)	64.2 (12.5) 85.3 (43.2)	62.2 (12.2) 91.2 (51.4)
Observed reflections^1^	89978 (4432)	54166 (2621)
Unique reflections^1^	26144 (1316)	15791 (790)
Average redundancy^1^	3.44 (3.38)	3.43 (3.32)
< I/σ(I)>^1^	4.6 (1.4)	4.2 (1.4)
R_meas_^1,2^	0.30 (1.14)	0.20 (0.65)
R_merge_^1,3^	0.25 (0.96)	0.17 (0.54)
CC_1/2_^1,4^	0.963 (0.553)	0.985 (0.756)
**Refinement**		
Resolution, refinement^1^(Å)	42.65-2.2 (2.27-2.22)	44.37-2.70 (2.77-2.70)
Rfree (5% set), Rwork^1^	0.257 (0.345), 0.193 (0.265)	0.234 (0.508), 0.187 (0.290)
Coordinate errors (free DPI, σ_A_), (Å)	0.341, 0.231	0.505, 0.372
F_o_ vs. F_c_ correlation, free	0.926, 0.876	0.923, 0.887
All refined non-H, *n*, <B> (Å^2^)	6871 (34.7)	6785 (32.0)
TLS groups	4 (1 for each molecule)	
OXL ligands	0	4 (1 per molecule)
Mg^2+^ cations	6 (1 per molecule + 2 intermolecular)	4 (1 per molecule)
K^+^ cations	0	2
Cl^−^ anions	6	9
Water molecules	120	35
**Geometry**		
r.m.s.d. bond lengths, angles (Å, °)	0.007, 1.47	0.007, 1.50
Ramachandran preferred, allowed, outliers^5^	789 (96%), 30 (4%), 0 (0%)	813 (95%), 42 (45%), 0 (0%)

* Image prefixes are: mesh, mesh scan images; line, the line scan images; ref, four characterization images (90 deg apart); the actual dataset image has no prefix.

^1^Values in parentheses are for the highest resolution shell.

^2,3^As defined in (International Union of Crystallography, 2012) [28].

^4^CC_1/2_ is Pearson’s correlation coefficient between two randomly assigned datasets each derived by averaging half of the observations for a given reflection as defined in (Karplus and Diederichs, 2012) [29].

^5^Determined using the Ramachandran plot boundaries defined in Molprobity (Chen et al., 2010) [30].

### Enzyme activity assay

ODx and ApH activities of recombinant mFAHD1 protein were tested via a defined 96-well plate assay, outlined in detail elsewhere [7]: buffer conditions were set to 50 mM Tris/HCl, 100 KCl, and 1 mM MgCl_2_ at pH 7.4. Sodium oxaloacetate (OAA) was bought from Sigma–Aldrich (HPLC grade, O4126), and acetylpyruvate was prepared via custom synthesis. Substrates were dissolved in assay buffer fresh at the start of each experiment (20 mM working solutions). Further dilutions were created to test different final substrate concentrations. In selected wells on a UV-transparent 96 well plate, increasing amounts (1–20 μg) of purified recombinant protein (>98%, after gel filtration) were dissolved in 95 μl of buffer, and incubated for 10 min at room temperature [7]. Asssociated blanks were created. Five microliters of substrate solution of increasing concentrations (adapted to the protein concentration) were added to the enzyme preparations and blank, to result in a final substrate concentration of 10 μM to 2 mM in 100 μl total volume per well [7]. The decrease in substrate concentration was observed at 255 nm wavelength via a plate reader at 25°C. Enzyme activity and kinetic profiles were obtained via the initial reaction rates and a non-linear least-square fit [7].

### Statistical analysis

Kinetic profiles of recombinant protein were obtained with three independent batches of protein preparations (*n*=3). Data analysis was performed using GraphPad Prism version 5 (www.graphpad.com). Presented data are the mean and standard deviation within 95% confidence interval.

### Antibodies

Polyclonal antisera against FAHD1 were raised against recombinant untagged hFAHD1 protein and His6/S-double-tagged mFAHD1 protein, both produced in *E. coli* [23]. Recombinant protein was purified from *E. coli* using a series of three subsequent chromatographic steps as described [7,23]. Approximately 4 mg of pure recombinant protein was used by a commercial supplier (Biogenes, Berlin, Germany) to produce specific antisera which were shipped to our laboratory. FAHD1-specific antibodies were obtained from raw sera by protein G affinity chromatography and gel filtration, followed by a second affinity purification using an affinity resin consisting of sepharose beads with immobilized purified antigen. Rabbit monoclonal anti-mouse FAHD1 antibodies, including RabMab 27-1 [23] were raised against affinity-purified recombinant mFAHD1 protein produced in *E. coli*. Four milligrams of purified His6/S-double-tagged mFAHD1 [7] were used by a commercial supplier (Epitomics Inc, Burlingame, U.S.A.) to produce several hybridoma clones, which were delivered to our lab. Best hybridoma clones were selected by a combination of ELISA and Western blot tests. Hybridoma clone 27-1 turned out to produce the most suitable antibodies and was expanded; antibodies were collected from the hybridoma supernatant and purified by protein G affinity chromatography and gel filtration.

### Western blot

SDS/PAGE was performed with 12.5% SDS polyacrylamide gels [7]. Western blot was performed with methanol activated PVDF membranes at 300 mA on ice for 1 h. Blocking was performed overnight with 5% skim milk PBS, including 1% Tween-20 (blocking buffer). After blocking, membranes were washed three times for 10 min with PBS, including 1% Tween-20. Primary antibodies against human and mouse FAHD1 (see section before) were diluted with blocking buffer to similar concentrations of 15 μg/ml, applied for 1 h. Membranes were again washed three times for 10 min with PBS, including 1% Tween-20. As both antibodies were raised in rabbit, the secondary antibody in use was Swine Anti-Rabbit Immunoglobulins/HRP (affinity isolated) P0399 by Dako, diluted 1:3000 in blocking buffer, applied for 30 min. Membranes were washed three times for 10 minutes with PBS, including 1% Tween-20, and two times for 10 min with PBS. Preheated Immobilon Western Chemiluminescent HRP Substrate (Millipore #WBKLS0500, Billerica, U.S.A.; 1+1 mixture of HRP Substrate Peroxide Solution and HRP Substrate Luminol Reagent) was applied for 3 min at room temperature in the dark. Membrane negatives were development via X-ray film (Fuji) in a dark chamber (X-ray film exposure for 10 s, fixation and development for 60 s).

### Antibody epitope mapping

To obtain five GFP-tagged protein fragments of mFAHD1 encoding consecutive regions of the protein (aa 1–51; aa 44–95; aa 88–139; aa 132–183; aa 176–227), ten primer pairs were designed: five GFP reverse primers with an overlapping region matching the 5′ end of the appropriate FAHD1 cDNA fragment and five FAHD1 forward primers with an overlapping region matching the 3′ end of the GFP cDNA.

**Table:** 

*GFP:*	*fwd*:	5′-GACTCGAGATGGTGAGCAAGGGCGAGG-3′
	*rev:*	5′-CTTTGGGTCATCTTGTACAGCTCGTCCATGC-3′
*GFP-FAHD1_1…51:*	*fwd:*	5′-AGCTGTACAAGATGACCCAAAGCTGTACTATGG-3′
	*rev:*	5′-GAGGATCCTCACGGCTTCAGGAAAAGCACAG-3′
*GFP-FAHD1_44…95:*	*fwd:*	5′-GCTGTACAAGGAGCCTGTGCTTTTCCTGAAG-3′
	*rev:*	5′-GAGGATCCTCAGTCCATGGCTGCAGCCTC-3′
*GFP-FAHD1_88…139:*	*fwd:*	5′-GCTGTACAAGATCCCGGAGGCTGCAGC-3′
	*rev:*	5′-GAGGATCCTCAGGGCACGAAGGCACTGAC-3′
*GFP-FAHD1_132…183:*	*fwd:*	5′-GCTGTACAAGTGCCCGGTCAGTGCCTTC-3′
	*rev:*	5′-GAGGATCCTCATATTATCTTAGAAACATAGCTGATGATG-3′
*GFP-FAHD1_176…227:*	*fwd:*	5′-GAGCTGTACAAGATCAGCTATGTTTCTAAG ATAATAACC-3′
	*rev:*	5′-GA-GGATCCTCAGTATTCTGATCTTTTCACCTTG-3′

The forward primer for the 5′ GFP sequence and the reverse primer for the different FAHD1 fragments were designed to contain a XhoI or BamHI restriction site, respectively. Full-length cDNA of mFahd1 and mGfp was used as template for the amplification via PCR. The expected size of the PCR products is 600 bp for Gfp and ∼150 bp for the Fahd1 fragments. After amplification of the mGfp and mFahd1 sequences each complimentary PCR product (FAHD1_1-5 and GFP_1-5) was fused together in an additional PCR, resulting in an 800-bp product due to annealing of the complementary overhangs. This reaction was carried out without any primers using standard PCR thermal cycling conditions with 10 cycles instead of 25. In the last step the GFP-FAHD1 fragments resulting from the sewing PCR were amplified using the forward primer for the 5′ GFP sequence and the appropriate FAHD1 reverse primer with a final standard PCR. The obtained PCR products encoding different GFP-tagged FAHD1 fragments were then transferred into the multiple cloning site of the eukaryotic expression vector pcDNA3.1(-) Hygro (Invitrogen). Both the purified PCR products as well as the vector were digested with BamHI and XhoI to generate sticky end overhangs, followed by dephosphorylation of the vector by adding 1 μl shrimp alkaline phosphatase for 1 h at 37°C. After ligation and transformation of chemically competent *E. coli* Top10 bacteria (Life Technologies), plasmid DNA was prepared from single colonies. Positive clones were identified by a restriction digest using XhoI and HindIII, resulting in 6000 bp (vector) and 800 bp (insert) fragments, and further verified by sequencing (Eurofins MWG Operon, Germany). To verify cloning of an insert into the recipient vector or to generate appropriate overhangs to ligate an insert into the vector DNA, fragments were digested by specific restriction endonucleases. The reaction mix was prepared as follows and incubated for 1 h at 37°C. To clone the digested insert into the pcDNA3.1/Hygro(-) vector, the complementary restriction fragments were fused with T_4_ DNA ligase. For the enzymatic reaction 60 ng of the linearized vector and a five-fold molar excess of the insert were mixed together with 2 μl of 10× ligase buffer and 1 μl (five units) T_4_ DNA ligase. The ligation mixture was incubated overnight at 16°C. Agarose gel electrophoresis is a simple method that allows the separation and purification of DNA fragments according to their size. A constant current of 80–100 V was applied until the samples were separated, and results were documented using a UV transilluminator (wavelength 254 nm). DNA of interest was recaptured from the gel and purified by using the QIAquick Gel Extraction Kit (Thermo Scientific) according to the manufacturer's protocol. DNA was eluted in a volume of 30 μl TE/H_2_O. Chemically competent *E. coli* Top Ten bacteria (Life Technologies) were thawed on ice and 1–100 ng plasmid DNA were mixed with 150 μl of cell suspension. After mixing the tube shortly by carefully tapping the tube, the mixture was incubated on ice for 30 min. Bacteria were heat-shocked for 30 s at 42°C to facilitate uptake of the plasmid into the cell and put back on ice for 2 min. A total of 250 μl of LB medium was added to the bacterial suspension and incubated at 37°C for 1 h while shaking; 100–150 μl of the transformation mixture was plated on to LB agar plates containing ampicillin for selection of successful transformed bacteria (the plasmid vector carries an ampicillin resistance gene). Plates were incubated overnight at 37°C. Single colonies were picked and transferred into 3 ml of LB medium supplemented with 100 μg/ml ampicillin followed by an incubation overnight at 37°C while shaking. This culture was used for further isolation of plasmid DNA.

## Results

### Structural comparison of hFAHD1 and mFAHD1

Using oxalate as competitive ODx inhibitor [6,7], complexed and native crystal structure models of recombinant mFAHD1 were obtained, and structure factors and refined structure models have been deposited with the PDB (6SBI, 6SBJ) (Table 1). Similar to the crystal structures of hFAHD1 (6FOG, 6FOH), *N*-terminal residues are disordered in both models, but ligand-associated conformational differences are present in the complexed structure [6] (Figure 1A), and are similar among the four proteins in the ASU. The chemical environment of the ligand-bound mFAHD1 cavity (Figure 1B) is similar to the hFAHD1 environment [6,7].

**Figure 1:** Structural comparison of native and complexed mFAHD1 (**A**) Root-mean-square-deviation (RMSD) between each of the proteins in the ASU in the native (6SBJ, red) and complexed (6SBI, black) structure. The average RMSD is below 0.25Å, except for five regions, denoted by their major peaks in the RMSD per residue plot. The major two regions are marked by color (red and blue), that map to (**B**) of this figure. The red region indicates the flexible ‘lid’ region of FAHD1, that rigidifies upon ligand binding. Amino acid residues 33–42 are missing in 6SBJ due to disorder and excluded from the plot. (B) Sketch of the mFAHD1active site (6SBI), in analogy to hFAHD1 (6FOG) [6]. The two regions around residues H33 to E36 (denoted in red), and around Q112 to K118 (denoted in blue) become ordered upon ligand binding. Compared with data presented in (A) with the same coloring.

The overall well-conserved sequences of mFAHD1 and hFAHD1 (Table 2, Figures 2A and 3A) differ at a total of 24 amino acid residues (Table 3 and Figure 3B). hFAHD1 (UniProt: Q6P587) is expressed in three isoforms, that differ in the *C*-terminus [2,3]. mFAHD1 (UniProt: Q8R0F8) is expressed in only one isoform [2,3], with highest sequence similarity to isoform 1 of the human protein (Figure 2B). The major secondary structure motifs are identical among the protein orthologs. The *N*-terminal ‘lid’-structure [6] in hFAHD1 in between G24 and E33 is also present in mFAHD1. The catalytic center, defined in the human protein by amino acid residues G24, R25, H30, E33, K47, E71, E73, D102, Q109, and K123, is also found in the mouse crystal structure with residues G27, R28, H33, E36, K50, E74, E76, D105, Q112, and K126 (Figure 1B). Correspondingly, human and mouse protein show similar Michaelis–Menten kinetics (Table 3 and Figure 4), and mFAHD1 displays the same bifunctionality as ODx and ApH. Despite the high level of overall structural similarity, 11 of the 24 residue substitutions cause significant changes in the side-chain chemistry of the protein (Table 3). Particularly affected is a surface-located sequence between amino acid V62 and A98 (mFAHD1 numbering), that involves a noticeable change in side-chain chemistry within a rather short peptide sequence. The structural differences in section V62 to A98 between mouse and hFAHD1 is displayed in Figure 5. Major changes in side-chain chemistry are observed in section L80 to E86 of the mouse protein, involving a change from M78 (human) to L81 (mouse), C82 (human) to G86 (mouse), and R83 (human) to E86 (mouse), therefore slightly decreasing the polarity of the local surface area of the mouse protein compared with the human, but also exchanging a positively charged arginine by a negatively charged glutamate residue.

**Figure 2:** Overall structural comparison and sequence alignment of hFAHD1 and mFAHD1 (**A**) Overlay and independent model structures of chain A in human (PDB: 6FOG) and mouse FAHD1 (PDB: 6SBI) after structural alignment. The general similarity is apparent, and further analysis (see Figure 3A), displays a low deviation among proteins in the unit cell. Sequence numbers in the aligned core proteins are offset by 3 due to the N-terminal differences. (**B**) Amino acid sequence alignment and comparison of human isoform 1 (UniProt: Q6P587) and mouse FAHD1 (UniProt: Q8R0F8). Boxes indicate differences in the amino acid sequences, as also listed in Table 3. Dark gray coloring thereby indicates changes in the chemical nature of the amino acid side chains.

**Figure 3:** Backbone root-mean-square-deviation between mFAHD1 and hFADH1 and side-chain differences (**A**) Plotted root-mean-square-deviation (RMSD) of backbone atomic positions, comparing mFAHD1 (PDB: 6SBI) with human FAHD1 (PDB: 6FOG), based on mean atom position of proteins in the ASU in each structure. The general RMSD is below 1.0 Å, with a set of 24 amino acid residues displaying slightly higher deviation in the backbone conformation (backbone defined via N-CA-C-O; data computed with UCSF Chimera [22]). The strongest outliers are labeled. Major side-chain differences are highlighted in (**B**). (B) Highlighted major changes in the chemical nature of the amino acid side chains. Blue structures correspond to chain A in hFAHD1 (PDB: 6FOG), and green structures display chain A in mFAHD1 (PDB: 6SBI) (see also Table 3). These differences are similar among proteins in the unit cell.

**Figure 4:** Michaelis–Menten kinetics of ODx and ApH activities of mFAHD1 (**A**) ODx activity of mFAHD1: within the accuracy of a photometric assay [7], v_max_ ranges from 0.18 to 0.24 μmol/min/mg, and *K*_M_ ranges from 8 to 78.0 μM, similar to hFAHD1 [6,23]. Within the given range, our best-model fit found v_max_ = 0.21 μmol/min/mg and *K*_M_ = 42.8 μM (see Table 2). Dashed lines correspond to the borders of the stated v_max_ ranges. (**B**) ApH activity of mFAHD1: within the accuracy of a photometric assay [7], v_max_ ranges from 0.13 to 0.16 μmol/min/mg, and *K*_M_ ranges from 3 to 11 μM, similar to hFAHD1 [6,24]. Within the given range, our best-model fit found v_max_ = 0.14 μmol/min/mg and *K*_M_ = 7.2 μM (see Table 2). Dashed lines correspond to the borders of the stated v_max_ ranges.

**Figure 5:** Structural differences in section V62 to A98 between mouse and human FAHD1 The structural differences in section V62 to A98 between mouse and hFAHD1 are indicated, displaying the plasticity within each ortholog. Each PDB entry (6FOG, 6SBI) has NCS tetramers per respective ASU. To illustrate this difference, as well as plasticity this figure displays a stick-model superposition of the region where the human structures superimposed are shown in blue and the mouse structures in green. A special highlight is given to the hypothesized epitope region in section L80 to E86 of the mouse protein.

**Table 2:** Comparison of FAHD1 in human and mouse

Properties	*human*^2^			*mouse*^2^
Number of isoforms	3			1
Number of amino acids	224	226	248	227
Molecular weight (Da)	24843	24910	27128	25172
Theoretical pI	6.96	7.64	7.60	7.58

Kinetic properties ODx	*human*^6^	*mouse (this work)*
k_cat_ (nmol/min/mg)	210 (196–230)	210 (181–239)
K_M_ (μM)	40 (24–57)	43 (8–78)

Kinetic properties ApH	*human*^6^	*mouse (this work)*
k_cat_ (nmol/min/mg)	140 (117–165)	140 (129–158)
K_M_ (μM)	5 (3–42)	7 (3–11)

**Table 3:** List of different residues comparing FAHD1 in human and mouse

*human*	*mouse*
A^6^-S^7^-R^8^	S^9^-T^10^-K^11^
R^32^	K^35^
**A^37^**	**T^40^**
I^59^	V^62^
**T^63^**	**C^68^**
L^72^	V^75^
**V^77^-M^78^**	**L^80^-L^81^**
**C^82^-R^83^**	**G^85^-E^86^**
V^85^	I^88^
G^95^	A^98^
D^110^	E^113^
**A^127^**	**S^130^**
**K^145^**	**A^148^**
K^147^	R^150^
**E^161^**	**K^164^**
I^187^	L^190^
V^199^	I^202^
**H^210^**	**D^213^**
L^212^	V^215^
**T^216^**	**R^219^**

### Generation and characterization of antibodies to mFAHD1

In collaboration with commercial suppliers, both polyclonal and monoclonal antibodies against mFAHD1 were generated based on full length mFAHD1 protein purified in our laboratory. Antibodies were tested for specificity and selectivity by Western blot. As expected, both rabbit monoclonal antibody (RabMab 27-1) and polyclonal rabbit antiserum raised against full-length mFAHD1 recognized the protein in lysates from heart, liver and kidney of wild-type mice, and no signal was obtained in spleen lysates (where FAHD1 is not expressed) and kidney lysates from Fahd1 KO mice, assessed as additional control (Figure 6A).

**Figure 6:** Identification of the epitope recognized by the monoclonal rabbit mFAHD1 (**A**) Thirty microgram protein isolated from mouse tissue lysates were analyzed by Western blot, using a polyclonal α-mFAHD1 antibody and RabMab 27-1 (see ‘Materials and methods’ section). Kidney lysate of an FAHD1 knockout mouse was used as negative control, α-TUBULIN antibody (Sigma–Aldrich) was used as loading control. Lower molecular weight signal detected by the polyclonal antibody (not displayed) are non-specific and the intensity of the specific signal is roughly comparable between polyclonal and monoclonal antibodies. (**B**) Full-length FAHD1 was divided into five different constructs, encoding consecutive regions of the protein (aa 1–51; aa 44–95; aa 88–139; aa 132–183; aa 176–227) which were fused with GFP. Protein lysates from U2OS cells transfected with pcDNA_3.1_GFP-FAHD1 plasmids 1–5 were analyzed by Western blot analysis using mFAHD1 antibody and antibody directed against GFP. U2OS cells transfected with pcDNA_3.1_Hygro (-) (empty vector) served as negative control and cells transfected with Fahd1 overexpression plasmid (FAHD1_OE) as positive control.

To address potential binding sites of RabMab 27-1 on mFAHD1, the cDNA of mFAHD1 was fused with the cDNA of green fluorescent protein GFP (see ‘Materials and methods’ section), and five overlapping GFP-tagged fragments of mFAHD1 were created, expressed in *E. coli*, and separated by SDS/PAGE (Figure 6B). The epitope region was narrowed down to a protein fragment ranging from amino acid E44 through D95.

### RabMab 27-1 detects a defined epitope on mFAHD1 that differs from hFAHD1

Surprisingly, RabMab 27-1, did not cross-react with hFAHD1 protein expressed in *E. coli*, whereas a rabbit polyclonal antiserum raised against hFAHD1 protein recognized both human and mouse proteins (Figure 7A).

**Figure 7:** RabMab 27-1 against a defined epitope does not recognize hFAHD1 (**A**) RabMab 27-1, raised against recombinant mFAHD1 was produced (see ‘Materials and methods’ section), that was found to recognize its antigen, but not hFAHD1. A Western blot (see ‘Materials and methods’ section) displays a clear differentiation with comparable concentrations of primary antibodies. Bands stem from the same gel and splice borders are indicated by the dashed line. Loaded FAHD1 was recombinant protein purified via His-tag and Ni-NTA affinity chromatography, following a defined protocol [7]. We find that both proteins display slightly different apparent protein masses on an SDS/PAGE gel. (**B**) Epitope analysis revealed that the region of interaction is situated in between amino acids 44 and 95 (Figure 6). Subsequent bioinformatics analysis, based on the available protein structures and sequences, suggest that the epitope is around the variant amino acid sequence L80 to I88 in mFAHD1 (V77 to I85 in hFAHD1), accounting for the major difference between the two structures.

To further address the precise position of the epitope on mFAHD1 recognized by RabMab 27-1, structural differences between mFAHD1 and hFAHD1 in the domain fragment ranging from amino acid E44 through D95 were taken into account. Based on the three-dimensional structure of this domain (Figure 7B), the most likely position of the epitope spans amino acid residues between V77 and I88, which is referred to as the epitope LLGKRGEAI below. This domain constitutes a surface region which differs significantly between both species (Figure 5), and maps to the section of major changes in side-chain chemistry found by comparing the structures of human and mouse protein.

Western blot data revealed that the polyclonal antibody produced in our laboratory recognized mFAHD1 in various tissues of wild-type but not Fahd1-KO mice, including liver, kidney, pancreas, and a few others (Figures 6 and 8B). RabMab 27-1, on the other hand, failed to recognize mFAHD1 in pancreas lysates of wild-type mice, although the protein is clearly expressed in this tissue and detected by rabbit polyclonal antibody to mFAHD1 (Figure 8B). These data suggest that the epitope LLGKRGEAI is not readily accessible in the majority of FAHD1 molecules from murine pancreas, raising the possibility that the epitope may be masked in this particular tissue, for example by a post-translational modification, such as acetylation. However, more work will be required to address this point. Of note, K83 in the center of this epitope section was recently reported as a SIRT3 deacetylation site [25], which will be further discussed below.

**Figure 8:** Lysine 83 in mFAHD1 is a reported SIRT3 deacetylation target (**A**) K83, K116, K117, and K142 of mFAHD1 have been reported to be deacetylation targets of SIRT3 [25]. K83 (K80 in hFAHD1) is in the center of the identified epitope region of the monoclonal antibody (Figure 7). The lysine side chain is depicted in green for both hFAHD1 and mFAHD1; residues comprising the putative epitope LLGKRGEAI in mouse FAHD1 are shown in red; the corresponding amino acid residues in hFAHD1 are depicted in blue. (**B**) Western blot of FAHD1 in an exemplary collection of mouse organs (wild-type and mFAHD1 knockout mice), similar to data presented elsewhere [23,24]. In contrast with the polyclonal antibody, RabMab 27-1 seems to be tissue specific, i.e., hindered in recognizing the antigen in certain tissues, such as pancreas (lowest plot, left subpanel). Western blot has been repeated three times (*n*=3), and the signals of polyclonal and monoclonal antibodies (normalized to the Tubulin signal) have been compared (right subpanel). Error bars represent the standard deviation within 95% confidence interval. We find that RabMab 27-1 recognized mFAHD1 in pancreas tissue, but the signals are significantly weaker than compared with kidney (*P < 0.05; P = 0.04).

## Discussion

FAHD1 was described previously as regulator of mitochondrial function and senescence [4,5]. According to our current hypothesis, FAHD1 as ODx is involved in the regulation of the TCA cycle flux, probably by regulating the activity of complex II (succinate dehydrogenase, SDH) in the respiratory chain via inhibition by OAA. In order to better understand the changes in metabolism and associated phenotypes in higher organisms, that may be induced upon FAHD1 regulation or mutation, current research aims for studies in a mouse model. We previously suggested that individual mechanisms of FAH superfamily enzymes are dictated by the orientation of the bound substrate in the cavity and the local destabilization by individual sidechains [6]. To support this research, FAHD1 proteins from human and mouse were compared in terms of structure and enzymatic activity.

We find that FAHD1 displays bifunctionality as ODx [23] and ApH [24] in both human and mouse with comparable kinetic profiles. This is understood by comparing the core structures, differing in only 24 amino acid residues and displaying the same secondary structure and an identical catalytic center. The catalytic mechanism [6] and metabolic function [23,24] are suggested to be identical in both organisms. Among the different residues, a sequence of 5 strongly varying surface located residues was identified, that may be used as epitope to produce of species-selective primary antibodies. Providing species-selective FAHD1 antibodies for proteomic approaches, histology and immune-fluorescence will further enable elaborate research on FAHD1 in the mouse model, which is certainly warranted. In addition, one future goal of this work will be the development of a reagent that may detect post-translational modifications of the FAHD1 protein, i.e., the K83 selective acetylation of mFAHD1.

Of note and interest, K83 of mFAHD1 is reported to be a deacetylation target for mitochondrial protein deacetylase SIRT3 [25], and we found this amino acid side chain to be located at an exposed position at the surface (Figure 8A). SIRT3 is emerging as a metabolic sensor that responds to changes in the energy status of the cell and modulates the activity of key metabolic enzymes via protein deacetylation. SIRT3 is localized to the mitochondrial matrix and its expression is selectively activated during fasting and calorie restriction [25]. In particular, SIRT3 is reported to regulate mouse pancreatic β-cell function [26], and to promote the urea cycle and fatty acid oxidation during dietary restriction [27]. Given that FAHD1 is a mitochondrial metabolic enzyme, SIRT3 targeting FAHD1 is a very interesting idea in order to elaborate our model.

Data comparing polyclonal and monoclonal antibodies indicates that the monoclonal antibody is somehow hindered to detect mFAHD1 in pancreas lysates by Western blot (Figure 8B). This observation supports our hypothesis of a definitive intrinsic difference between the mouse and human FAHD1 polypeptide chains, which cannot be explained by epitope masking, due to differential protein folding or steric inhibition of antibody access by a putative interaction partner. Combining these data, we hypothesize that acetylation of surface exposed K83 of mFAHD1 could interfere with the binding of the monoclonal antibody. If this is true, our antibody could be used as a tool for the detection of SIRT3-specific acetylation states of the mFAHD1 protein, and potentially as a marker for mFAHD1 regulation during aging.

Given that mitochondrial dysfunction can induce a spectrum of senescence-like phenotypes [5], and that FAHD1 is involved in the regulation of the TCA cycle flux [6], understanding mFAHD1 in an *in vivo* model will contribute to the understanding of the underlying physiological or pathological process of FAHD1 deregulation. We have initiated *in vivo* studies with mFahd1 knockout in a mouse model, that will provide insight into potential phenotypes associated with the absence of mFAHD1, about which we will report in due time. Present data, showing that FAHD1 displays comparable structure and function in human and mouse, represent an essential step to enable for associating results of such studies with comparable human phenotypes.

## Abbreviations

ApH: acylpyruvate hydrolase
ASU: asymmetric unit
ESRF: European Synchrotron Radiation Facility
FAH: fumarylacetoacetate hydrolase
FAHD1: FAH domain-containing protein 1
hFAHD1: human FAHD1 protein
KO: homozygous knockout of a gene
mFAHD1: mouse FAHD1 protein
NZCYM: medium used for cultivating recombinant strains of Escherichia coli
ODx: oxaloacetate decarboxylase
RabMab: rabbit monoclonal antibody
SEC: size exclusion chromatography
SIRT3: NAD-dependent deacetylase sirtuin-3, mitochondrial
TCA cycle: tricarboxylic acid cycle; Krebs cycle
TLS: Translation-Libration-Screw-rotation
